The article "Application of Digital Orthopedic Technology in Orthopedic Trauma" was retracted in 2023. Reasons: signs of a paper mill; suspected computer-generated content; unreliable results or conclusions; lack of ethics approval or compliance.

# Application of Digital Orthopedic Technology in Orthopedic Trauma

**DOI:** 10.1155/2022/3157107

**Published:** 2022-08-16

**Authors:** Jiangtao Lin, Junbo Ge, Jinpeng Gong, Huanyu Hong, Chuanqiang Jiang

**Affiliations:** The First Ward of Trauma Orthopedics, Yantaishan Hospital, Yantai 264003, China

## Abstract

In order to solve the limitation of auxiliary treatment means in the process of orthopedic trauma surgery, and further improve the effective integration of orthopedic trauma clinical surgery and computer technology, a new orthopedic trauma auxiliary treatment means based on digital orthopedic technology was proposed with the aid of virtual digital technology. The method builds a 3D model of fracture fragments through 3D orthopedic modeling and obtains a high-quality 3D model through processing. Later clinical tests verify the feasibility of this auxiliary treatment method. The test results show that the precision of the 3D reconstruction model based on custom option fitting is higher than that based on optimal option fitting, and the precision difference is within 0.2%. This result also indicates that the 3D model obtained by 3D reconstruction has higher accuracy. The results show that three-dimensional finite element modeling technology can accurately simulate the stress of the spine of orthopedic patients and can reduce the incidence of complications through preoperative diagnosis, curative effect prediction, and trauma surgery, which has a good aid for postoperative recovery.

## 1. Introduction

In recent years, with the rapid development of digital technology, it provides a new technical means for the basic research of clinical treatment of orthopedic diseases, especially through the mutual integration and mutual influence of traditional orthopedic theory, gradually forming a modern digital orthopedic treatment technology with digital characteristics. At present, the techniques applied in orthopedic surgery mainly include medical image processing and 3D modeling, 3D virtual simulation and visualization, computer-aided design, finite element technology, mechanical simulation of human skeletal muscle system in robot-assisted treatment, etc. These techniques have greatly improved the therapeutic effect and technical level of orthopedic surgery. As a special type of orthopedics, traumatic orthopedics has different characteristics from spinal surgery and joint surgery, and the integration of digital technology and traumatic orthopedics is becoming more and more extensive. In this study, higher quality 3D models were obtained by constructing 3D orthopedic models. With the support of 3D finite element modeling technology, the feasibility of digital orthopedic-assisted therapy was verified through clinical tests.

The article "Application of Digital Orthopedic Technology in Orthopedic Trauma" was retracted in 2023. Reasons: signs of a paper mill; suspected computer-generated content; unreliable results or conclusions; lack of ethics approval or compliance.

## 2. Literature Review

Yang and others say that in traditional orthopedic research, surgeons have to rely solely on images of patients to determine surgical procedures in their heads [1]. Wang et al. say that the advantages of digital orthopedic techniques over traditional orthopedic models lie in preoperative planning for a three-dimensional anatomical model of the site. The 3D model of the affected area was printed by 3D and the operation was simulated directly [2]. Wang et al. say that finite element analysis can provide biomechanical support for surgical protocols [3]. Back and Pfrringer said that foreign studies include the following: in a proposed train-oriented simulation framework for temporal bone surgery, the system allows two users to observe and operate a common model in different locations to perform an operation and allows each user to experience the influence of the force generated by the contact of other users with the bone surface [4]. Adam and others say the system also allows teachers to observe students remotely and provide real-time feedback and demonstrations. Virtual reality software and workflow applications were used for radiotherapy, treatment planning, and evaluation using virtual linear accelerators [5]. The result is that it is possible to simulate most radiotherapy workflows and tasks. Rawal and others say the method saves time and is relatively safe, allowing for a good understanding and experience of clinical procedures in advance. A new haptic surgical simulator for cerebral aneurysms was developed, and its role in neurosurgical residency training was evaluated [6]. Stogov et al. say that surgical treatment of cerebral aneurysms is complex and rare and that a simulation-based tool is needed to educate future neurosurgeons to operate on cerebral arteries [7]. The simulator is a virtual reality aneurysm surgery simulator based on real-time haptic feedback. It adopts an immersive touch platform to provide aneurysm and vessel volume deformation and aneurysm rupture during surgery with haptic feedback. Ow et al. said that 17 neurosurgeons who tested the simulator in three ways said it was very similar to actual aneurysm surgery [8]. Doctors believe that the simulator provides immersive anatomical details for surgical dissection and accurate guidance and is useful for preoperative surgical practice and neurosurgical training. Hamsen and others say that 3D printing is based on digital model files, which use adhesive materials such as powdered metal or plastic to print layer by layer until the desired object is constructed. It is a digital technology [9]. 3D printing technology can provide a more complete personalized solution for the medical industry. Typical applications include 3D printing of preoperative planning models, surgical guides, prosthetic implants, and medical rehabilitation instruments such as hearing aids. Good preoperative planning is the key to successful operation. In particular, for difficult and high-risk operations or new operations, preoperative planning is particularly important. Compared to 2D data, 3D data is more realistic, and the 3D model is printed by a 3D printer. It can not only assist doctors to carry out accurate surgical planning and formulate more accurate and detailed surgical plans to improve the success rate of surgery but also facilitate doctors to have better intuitive communication with patients and their families on surgical plans. Hang and others say biomedical 3D printing in China, while still in its infancy, is becoming more widely used. Due to the individual characteristics of different patients, preoperative simulation can be customized, and the customized characteristics of 3D printing technology bring great convenience to personalized treatment. Academician Dai Zhirong believes that 3D printing technology has brought good news to the medical field (see [10]). Taking orthopedic implants as an example, complex porous structures integrated with the implants can be directly printed on the surface of the implants by 3D printing technology. These structures are conducive to bone growth and patient rehabilitation. Denture processing, for example, allows dental scanners and 3D printers to print denture models of multiple patients at the same time, freeing dentists from the role of artisans making plaster casts by hand and freeing them up to spend precious time on treatment. Take surgery, for example, by combining medical image data design software with 3D printing, doctors can not only see a three-dimensional model of the patient on a computer but also 3D print the model and use the physical model for precise surgical planning and practice. It can help doctors develop a more accurate surgical plan; thus, the operation time is shortened and the success rate of the operation is improved. For the clinical treatment of developmental hip dysplasia (DDH), 3D printing technology was used to print the lesion models of 10 patients with DDH. Computer-aided measurement was used to simulate the operation, measure the size of the used prosthesis, and compare it with the actual postoperative value. The results showed that there was no significant difference between the measured values of acetabular diameter lines and the actual values, the acetabular rotation center was found accurately, and the use of the prosthesis was consistent with the preoperative plan. In the 3D printing group, intraoperative blood loss, operative time, postoperative drainage, postoperative complication rate, and so on were better than those of conventional surgery. 3D printing technology can improve the precision and efficacy of DDH joint replacement surgery. China's first 3D-printed orthopedic implant 3D-printed artificial hip product applied by Peking University Third Hospital, one of the supporting units of the TCT Asian exhibition, has been approved by the State Food and Drug Administration. The Third Affiliated Hospital of Southern Medical University (Guangdong Orthopaedic Hospital) carried out the first 3D-printed artificial vertebra implantation operation in Guangdong Province, successfully implanted the 3D-printed artificial vertebra in a patient with chordoma. Kang Yujian, an academician of the American Academy of Toxicology, said that 3D printing has changed the traditional medical operation mode and realized customized medical precision medicine, which means that customized health is no longer far away from us. The application of digital orthopedic technology in orthopedic trauma is shown in Figure 1.

The article "Application of Digital Orthopedic Technology in Orthopedic Trauma" was retracted in 2023. Reasons: signs of a paper mill; suspected computer-generated content; unreliable results or conclusions; lack of ethics approval or compliance.

## 3. Method

The finite element method regards the whole structure as a geometric entity connected by finite elements, and the assembly effect of the mechanical characteristics of each small element reflects the overall mechanical properties of the structure. The finite element analysis process is composed of algebraic equations to solve a series of problems, as shown in the following formula:

(1) $$\begin{array}{c} \left[K\right]\left\{U\right\}=\left\{Q\right\}. \end{array}$$

The finite element analysis process is composed of algebraic equations to solve a series of problems, as shown in Formula (1).

These quantities are indeterminate and are described quantitatively depending on the problem to be solved. The theoretical stress analysis is to analyze the stress distribution by mathematical models, while the finite element method is to divide the elements. It simulates the real structure to some extent and describes all aspects of the structure numerically. The accuracy of its description depends on the degree of unit subdivision, often based on experimental data. In the process of solving the problem, the structure description is combined with the algebraic equation of solid mechanics theory to find the stress and displacement of the required solution. The application process of the finite element method includes the following three main parts: data input, operation, and data output [11].

*Adaptability to complex geometric configurations*: a unit can be one-dimensional, two-dimensional, or three-dimensional in space, and each kind of unit can have a different shape, for example, a three-dimensional unit can be tetrahedral pentahedron or hexahedron. At the same time, different connection methods can be adopted between various elements. For example, the field function can be kept continuous between two surfaces, the derivative of the field function can also be kept continuous, or only the normal component of the field function can be kept continuous. *Applicability to various physical problems*: since the unknown field functions in the whole solution domain are represented by fragments of approximate functions in cells, there is no restriction on the form of equations that the field functions satisfy, nor on the same form of equations corresponding to each cell. Therefore, although the finite element method was initially proposed for linear elastic stress analysis, it soon developed elastoplastic problems, viscoelastoplastic problems, dynamic problems, buckling problems, etc. [12].

The article "Application of Digital Orthopedic Technology in Orthopedic Trauma" was retracted in 2023. Reasons: signs of a paper mill; suspected computer-generated content; unreliable results or conclusions; lack of ethics approval or compliance.

On the basis of previous studies, some scholars proposed to establish a three-dimensional model of implant-bone interface by using microscopic slices. The advantage of this method is that the thickness of the section is uniform, and the bone density and interface bonding of the trabecular bone can be reflected. The data are accurate and reliable. The disadvantages are that it takes a long time to complete, and it takes 2 months to process an implant image. The modeling methods of the finite element method can be the grinding disc method and CT scanning tomography, and their characteristics are shown in Table 1.

Load has three elements: size direction and point of operation. A static load is a load that increases gradually from zero to a final value with little or no change. The load that does not meet the static load condition is called a dynamic load. Under the dynamic load, the component produces an acceleration field which cannot be neglected [13, 14]. The dynamic load can be divided into inertial force and impact load; the latter is closely related to oral biomechanics. The relation between impact load and static load is shown in the following formula:

(2) $$\begin{array}{c} P_{d}=KP. \end{array}$$

*P*_*d*_ is the impact load, *P* is the static load, and *K* is the impact dynamic load coefficient.

*E*_*f*_ and *μ*_*f*_ are set as the elastic modulus and Pearson's ratio of the femur of knee joint occlusal elastomer, respectively. Here,*f*represents the femur, and*E*_*i*_and*μ*_*i*_represent the elastic modulus and Pearson's ratio of the tibia of knee joint occlusal elastomer, respectively. Here, *t* represents the tibia, and *R*_*f*_ and *R*_*f*_′ are two principal curvature semimeridions of the contact surface of the elastic femur occlusal. *R*_*t*_ and *R*_*t*_′, respectively, are the two principal radii of curvature of the contact surface of the tibial occlusal of elastomer. *a* and *b*, respectively, are the major semiaxis and the minor semiaxis of the elastic contact surface of the tibial joint of the knee joint. *δ* is the relative displacement of the elastic center of femur and tibia, *q*_0_ is the maximum compressive stress of the elastic contact surface of tibial articulation of the knee joint, and *P* is the axial static pressure. Thus, according to the Hertz theory, the fixed solution of the maximum compressive stress elastic contact area and deformation of the articulation contact area of the knee joint can be deduced, as shown in the following formula:

(3) $$\begin{array}{c} q_{0}=\frac{3P}{2\pi ab}. \end{array}$$

The maximum compressive stress occurs in the center of the contact surface. As can be seen from the above equation, the maximum compressive stress is 1.5 times of the average compressive stress on the elastic contact surface of the tibial articulatory joint of the knee joint. To calculate this compressive stress, two half axes *a* and *b* in the elliptic contact area of the knee joint must be worked out first, and the derivation results are shown in the following formulas:

(4) $$\begin{array}{c} a=\partial \sqrt[{3}]{\frac{3}{4}\frac{P}{A}\left(\frac{1-\mu_{f}^{2}}{E_{f}}+\frac{1-\mu_{t}^{2}}{E_{t}}\right)}, \end{array}$$

(5) $$\begin{array}{c} b=\beta \sqrt[{3}]{\frac{3}{4}\frac{P}{A}\left(\frac{1-\mu_{f}^{2}}{E_{f}}+\frac{1-\mu_{t}^{2}}{E_{t}}\right)}, \end{array}$$

(6) $$\begin{array}{c} \delta =\lambda \sqrt[{3}]{\frac{9}{128}{AP}^{2}\left(\frac{1-\mu_{f}^{2}}{E_{f}}+\frac{1-\mu_{t}^{2}}{E_{t}}\right)}. \end{array}$$

Here is shown in the following formulas:

(7) $$\begin{array}{c} A=\frac{1}{2}\left(\frac{1}{R_{f}}+\frac{1}{R_{f}^{\prime }}+\frac{1}{R_{t}}+\frac{1}{R_{t}^{\prime \prime }}\right), \end{array}$$

(8) $$\begin{array}{c} B=\frac{1}{2}{\left[{\left(\frac{1}{R_{f}}-\frac{1}{R_{f}^{\prime }}\right)}^{2}+{\left(\frac{1}{R_{t}}-\frac{1}{R_{t}^{\prime }}\right)}^{2}+2\left(\frac{1}{R_{f}}-\frac{1}{R_{f}^{\prime }}\right)\left(\frac{1}{R_{t}}-\frac{1}{R_{t}^{\prime }}\right)\cos2\Phi \right]}^{1/2}, \end{array}$$

(9) $$\begin{array}{c} \cos\theta =\frac{B}{A}. \end{array}$$

*Φ* is the included angle between *R*_*f*_ and *R*_*t*_, the plane where the two main radii of curvature are located; *α*, *β*, and *λ* are the coefficients; and the value of *θ* can be calculated according to Formula (9) and obtained by referring to the table.

The article "Application of Digital Orthopedic Technology in Orthopedic Trauma" was retracted in 2023. Reasons: signs of a paper mill; suspected computer-generated content; unreliable results or conclusions; lack of ethics approval or compliance.

### 3.1. Mathematical Description of Elastic Occlusal Surface of Knee Joint

Since it is still difficult to establish a network for the accurate mathematical description of the real 3D articulation surface of the knee joint, polynomial numerical approximation is used to describe the femoral surface and tibial surface of the knee joint elastic occlusion. Assuming that both surfaces are continuous and smooth functions, they can be expressed in polynomial form as follows.

For the tibial occlusal surface, it is shown in the following formula:

(10) $$\begin{array}{c} f_{T}\left(x,y,z\right)={xe}_{x}+y\left(x,z\right)e_{y}+{ze}_{z}. \end{array}$$

*T* is the tibial surface, as shown in the following formula:

(11) $$\begin{array}{c} x,y=y\left(x,z\right),z. \end{array}$$

The above formula is the coordinates of points on the tibial occlusal surface, and *y* can be obtained through multiple approximation as shown in the following formula:

(12) $$\begin{array}{c} y=y\left(x,z\right)=\overset{n}{\underset{i=0}{\sum }}\overset{n-1}{\underset{j=0}{\sum }}a_{ij}x^{i}z^{j}. \end{array}$$

In the above formula, *a*_*ij*_ can be determined by the following least square method as shown in the following formula:

(13) $$\begin{array}{c} \overset{m}{\underset{r=1}{\sum }}{\left\{y_{r}-y\left(x_{r},z_{r}\right)\right\}}^{2}=\overset{m}{\underset{r=1}{\sum }}{\left\{y_{r}-\overset{n}{\underset{i=0}{\sum }}\overset{n-1}{\underset{j=0}{\sum }}a_{ij}x_{r}^{i}z_{r}^{j}\right\}}^{2}. \end{array}$$

It is shown in the following formula:

(14) $$\begin{array}{c} r=r\left(x_{r},y_{r}z_{r}\right). \end{array}$$

The above formula is the coordinate of measuring point *r* of the tibial occlusal surface, while *m* is the number of points measured by the tibial occlusal surface.

In the same way, the femur surface equation of knee elastic occlusion can be determined as shown in the following formula:

(15) $$\begin{array}{c} f_{F}\left(x^{\prime },y^{\prime },z^{\prime }\right)={x^{\prime }e^{\prime }}_{x}+y^{\prime }\left(x^{\prime },z^{\prime }\right)e_{y}^{\prime }+z^{\prime }e^{\prime }z. \end{array}$$

Combined with formulas (12)–(15), it can be seen that the accuracy of the two surfaces of knee elastic occlusal contact, namely, tibial occlusal surface and femur occlusal surface, depends on the number of corresponding measurement points and the number of polynomial items selected.

The object of the study was fresh sheep femur, which was selected because it was widely available and easily accessible. In the smooth middle section of the femur of the fresh sheep, the length was 50 mm, and two through holes with diameters of 5 mm were made for calibration. The purpose of doing this is as follows: first, it is relatively easy to carry out CMM for the smooth femur segment of sheep; second, a reference is established after calibration to ensure the accuracy of comparison.

The article "Application of Digital Orthopedic Technology in Orthopedic Trauma" was retracted in 2023. Reasons: signs of a paper mill; suspected computer-generated content; unreliable results or conclusions; lack of ethics approval or compliance.

### 3.2. Three-Dimensional Reconstruction of Sheep Femur from CT Scan

Mask 1 of sheep femur with CT scan interval of 0.6 mm was extracted from Mimics16.0, namely, the initial mask. The initial mask is copied and edited to obtain the mask of the calibration segment, that is, the processed mask. Then, select Calculate 3D option and reconstruct the 3D reconstruction model with initial mask processing. The same method was used to compare contours under different fitting options, and the polar coordinate gap (d/mm) was outputted to sort out the data. Shown in Tables 2–8 are the polar coordinate gaps of different contours under different fitting options.

The corresponding histogram of the sheep femur contour at different heights can be found in that when the fitting option is High Medium, the corresponding point difference of the sheep femur 3D reconstruction model is significantly greater than when the fitting option is Optimal Custom. When the fitting option was Optimal, the corresponding point gap of the sheep femur 3D reconstruction model was close to that of the sheep femur 3D reconstruction model when the fitting option was Custom. The accuracy of the 3D reconstruction model of fresh sheep femur was defined as follows: the percentage of the polar coordinate difference (d/mm) and the corresponding polar coordinate (D/mm) of the corresponding points.

Combined with the above table, the d/mm histogram of the polar coordinate distance at different heights under different fitting options is presented for intuitive observation as shown in Figure 2.

The load deformation generated after the cylinder compression test is shown in Figure 3.

By analyzing the above two tables and Figures 2 and 3, it can be seen that the quality of the 3D model is Optimal > High > Medium, and the minimum accuracy of the 3D reconstruction model of sheep femur fitted by the Optimal option is 4.208%, which is within an acceptable range due to the particularity of the skeleton. The 3D reconstruction model of sheep femur fitted by the Optimal option is 2.0% larger than that of fresh sheep femur, that is, about 0.16 mm. The CT scan data of fresh sheep femur used in this study have high pixels, and the 3D reconstruction model precision fitted by the Custom option is higher than that fitted by the Optimal option; the difference is within 0.2%. This means that the quality of the CT scan data is good. The 3D model obtained by 3D reconstruction based on the gray value has higher accuracy. Considering that the running speed and storage space of the computer and the accuracy difference between the two is within 0.2%, 3D reconstruction based on Contour is a better comprehensive consideration and the Optimal fitting method is superior Custom Indicates the fitting method.

The article "Application of Digital Orthopedic Technology in Orthopedic Trauma" was retracted in 2023. Reasons: signs of a paper mill; suspected computer-generated content; unreliable results or conclusions; lack of ethics approval or compliance.

## 4. Experiments and Analysis

Here, Mimics software is used to build a Pilon fracture 3D model through Pilon fracture CT data, demonstrating the specific steps of model building, reflecting the unique characteristics and advantages of digital orthopedics, and demonstrating its application value in clinical orthopedics. At the same time, the Pilon fracture was classified on the generated 3D model and compared with its own X-ray film to verify the accuracy of the X-ray film diagnosis [15]. The technical route is shown in Figure 4.

Mimics16.0 was imported into the DICOM medical image and Thresholding-Bone (CT) option. Due to the different gray values of the bone and soft tissue, the two can be separated and the ankle initial mask can be obtained through Region Growing. Then, the discrete elements were accurately separated by the Region Growing option, and the foot bone mask was obtained through which to reconstruct the overall 3D model of the initial foot and ankle fractures [16, 17].

In the preoperative simulation, it is essential to effectively separate the fracture fragments from the fracture. It is crucial to separate fracture fragments accurately. Because the fragments are in contact with each other and overlap, the surgeon needs to be involved in this stage to ensure that the fragments are separated correctly. The process of separating the boundary of the fracture fragment is the process of carefully editing each layer mask of the fragment. After correctly separating the first fracture fragment, Boolean Operations can quickly and accurately separate the remaining bone fragment. According to the above method, all the fracture fragments were separated in turn, including the parts without fracture such as the foot scaphoid. Since preoperative simulation was not affected, it was possible to complete the separation of the mask of each fracture fragment without separating it and then establish a 3D model with Calculate 3D-Optimal and use different colors to represent each fracture fragment for convenient observation [18].

Due to the cancellous bone structure in the distal tibia bone, there are many honeycomb holes in the reconstructed 3D model. The large number of holes increases the number of features in the 3D model and complicates the model. In the process of preoperative simulation, the holes in the 3D model will not affect the accuracy of preoperative simulation but will occupy a large amount of computer memory [19, 20]. In the process of the 3D printing model, the complexity of the 3D model makes it more difficult to print data, and the internal holes will generate redundant support and materials cannot be processed in the printing process, which increases the difficulty of 3D printing. To improve the model quality, the reconstructed 3D model is outputted as an STL file and imported into Geomagic Studio to process each fracture fragment model.

The article "Application of Digital Orthopedic Technology in Orthopedic Trauma" was retracted in 2023. Reasons: signs of a paper mill; suspected computer-generated content; unreliable results or conclusions; lack of ethics approval or compliance.

The VR operating system includes hardware devices and software devices, as shown in Figure 5.

Mapping tools are used such as a steel ruler vernier caliper and caliper inside and outside, according to the real object for reverse modeling, in UG to build a pedicle screw (6.5 mm × 45 mm), crosslink interbody fusion device (length 22 mm × width 10 mm × high 12 mm), 3D model, and simplified model. Pedicle screw interbody fusion devices are all produced by the Beijing Riebel Company [21]. The actual pedicle screw structure is complex, with many threads and tightening devices. These structures are not the focus of biomechanical analysis but will greatly increase the workload of finite element analysis, which is prone to collapse of finite element analysis or nonconvergence of results. Therefore, it is necessary to simplify the model of interbody fusion screw rod system.

The total spinal data of a 41-year-old normal male (scanning parameters: 120 kV, 166 mAs, layer thickness: 0.8 mm) were scanned by the SOMATOM Definition dual-source, CT machine, row 64, manufactured by Siemens in Germany. The CT data were imported into the Mimics software in DICOM format, and the vertebral body boundary was accurately differentiated and separated manually in the image processing stage. The method was the same as the Pilon fracture treatment in the previous chapter, and the single vertebral body spinal model of the C7-S1 segment was extracted, which was convenient for subsequent three-dimensional reconstruction, and the three-dimensional spinal model was obtained [22].

In finite element analysis, the quality and quantity of the mesh directly affect the accuracy of calculation results and solving time. In general, the more the number of mesh (mesh) with a higher density, the greater the precision of the results of the analysis, but eventually, at the same time, the solving time will increase; to solve the problem, the equipment, such as computers, will require higher performance requirements, so the correct selection of meshing quantity can better coordinate calculation accuracy and computation time, both to achieve the optimum [23, 24].

Figure 3 shows the relationship between solution accuracy (*u*), calculation time (*t*), and mesh number (*n*) in finite element analysis. Curve 1 shows the relationship between the solution accuracy (*u*) and the number of meshing (*n*). It can be seen from curve 1 that, within a certain range of solution accuracy, the solution accuracy increases significantly with the increase of meshing density, namely, the increase of the meshing number. However, in the second half of curve 1, it can be seen that the curve has a very flat trend, and the solution accuracy can be obtained beyond a certain range. As the number of grids continues to increase, the solution accuracy will hardly change; curve 2 shows the relationship between the calculation time (*t*) and the number of meshing (*n*). In a certain solution time interval, the solution time does not change significantly with the increase of the number of meshing. For example, when the first half of curve 2 exceeds a certain solution time, the solution time increases rapidly with the continuous increase of the number of grids, and the second half of curve 2 becomes steeper. Meanwhile, the performance configuration requirements of the solver computer also increase greatly.

The article "Application of Digital Orthopedic Technology in Orthopedic Trauma" was retracted in 2023. Reasons: signs of a paper mill; suspected computer-generated content; unreliable results or conclusions; lack of ethics approval or compliance.

The selection of mesh size is also an important factor affecting the solution accuracy in the later stage. Generally speaking, for simple statics analysis, if we pay more attention to the solution results of displacement variation, the finite element mesh can be divided into larger ones. The same solution model can divide different grid sizes for different structures according to different demands. For nonconcerned structures, the grid size can be appropriately larger, such as the vertebral structure in the spin-rod system in this study. As stress is emphasized in this paper, the grid control of the displacement structure should be smaller, such as the pedicle screw of the spin-rod system. Meanwhile, the specific grid size can also be set by referring to previous literatures with the same structure and verified solution results [25, 26].

In the process of finite element analysis, material properties have a great influence on the accuracy of analysis results. Many researchers outside China have proposed many reliable methods for human bone attachment materials. Among them, DICOM data and gray scale assignment is the most common one. The material process is completed in the FEA module of Mimics software [27]. In this finite element analysis of human spinal interbody fusion screw system, the gray value material assigning method was used to assign materials to open the model in Mimics software, and materials were attached in the FEA module. The parameters are shown in Table 9.

The article "Application of Digital Orthopedic Technology in Orthopedic Trauma" was retracted in 2023. Reasons: signs of a paper mill; suspected computer-generated content; unreliable results or conclusions; lack of ethics approval or compliance.

The interbody fusion screw rod system includes the pedicle screw crosslinking device, which is made of medical titanium alloy (Ti-6Al-4V). The material of the interbody fusion device is PEEK (polyetheretherketone), as shown in Table 10.

Among them, the mask of each vertebral body of the human spine is attached with material according to the gray value, and the nail bar system of intervertebral fusion is attached with a single material by the three-dimensional model.

Select Supports>Fixed Supports from the menu of Supports>Fixed Supports under the Static Structural environment, light the Face option, select the lower surface of the sacrum of each set of models, and fix it to ANSYS. The static analysis of Workbench 15.0 provides five common contact types, which are summarized in Table 11.

The finite element model established in this study simulated the stress state of the vertebral disc screw system in the standing posture of the human body. The trend was close to the actual stress in the standing posture of the human body. Qian et al. believed that the gravity line of the human body passed through the 7th cervical vertebra, the 1st lumbar vertebra, and the 1st sacral vertebra in the upright posture. According to the study by Pierre et al., the gravity line of the human body varies widely due to individual differences and does not completely coincide with the plumb line of cervical vertebra 7. Generally speaking, the gravity line of young people is generally behind, while the gravity line of older people is slightly ahead. According to the above theory, we assumed that the gravity line passed through the 7th cervical vertebra and applied a load of 500 N perpendicular to the ground on the 7th cervical vertebra, so as to simulate the gravity line when normal people stand as much as possible, and then calculated the force on the spine and the stress changes of different interbody fusion materials. The force on the spine is obviously different with the human posture. After loading 500 N force on the back of the cervical 7 spine in the four groups to simulate the normal human gravity line, the stress of the interbody fusion material in the whole and lumbar 2-lumbar 5 spine screw system was analyzed [28].

*Equivalent compressive stress of the l4-l5 vertebral body-combined screw rod system*: the maximum compressive stress of model A, model B, and model C was all in the pedicle of L5—A: 188.24 MPa, B: 184.76 MPa, and C: 187.03 MPa, respectively; in model D, the maximum compressive stress is in the connecting rod part, which is much larger than the first three groups, at 348.19 MPa.

The maximum compressive stresses of the nail rod system are all in front of the connecting rod—model A: 36.43 MPa; model B: 21.81 MPa; model C: 33.48 MPa; and model D goes up to 348.19 MPa.

The article "Application of Digital Orthopedic Technology in Orthopedic Trauma" was retracted in 2023. Reasons: signs of a paper mill; suspected computer-generated content; unreliable results or conclusions; lack of ethics approval or compliance.

The equivalent compressive stress between waist 4 and waist 5 is as follows: model A is basically distributed in the rear of the annulus fibrosus, and the maximum compressive stress is 0.92 MPa. The maximum compressive stress of model B and model C is at the back of the fusion material—model B: 6.31 MPa; model C: 73.35 MPa. The stress value of the intervertebral body is less than the limit stress of the corresponding material, and the effective strength support can be achieved within the online elastic range. The maximum compressive stress of lumbar 2/3 and 3 and 4 intervertebral discs was 2.57 MPa and 4.91 MPa, respectively. The maximum compressive stress in the third lumbar spine was 3.62 MPa at the posterior edge of the vertebral body, and the maximum compressive stress in the fourth lumbar spine was 19.71 MPa around the pedicle.

The maximum compressive stresses in model A, model B, and model C were all located at the pedicle of L5 with similar values, while the maximum compressive stress in model D was located at the lumbar connecting rod, which largely indicated that a large part of compressive stress after l4/5 fusion was transmitted to L5 through the bilateral connecting rod in the upright state. On the pedicle of the vertebral body, the conduction force through the vertebral body was reduced compared with that without surgery. The working compressive stresses of the screw rod system in model A, model B, and model C were all small and close in value, which was much smaller than that in model D with blank intervertebral space, indicating that most of the loads in the first three models were dispersed and transmitted through the annulus fibrosus nucleus pulposus bone crusher and PEEK fusion device. Although the maximum compressive stress of the intervertebral section in the first three models is different, the load through the intervertebral material conduction is not different in general. In this chapter, DICOM medical images were used to establish four groups of finite element models of human vertebra-interbody fusion screw rod system for different materials used in posterior lumbar surgery, and stress changes of different materials used in human spine were analyzed under standing posture and compared with normal the human body. The following conclusions were drawn:

1. The three-dimensional finite element method is used to model the force applied in the direction of gravity and calculate the force on the normal spine
2. Pure spinous process lamina can be used to achieve effective mechanical support in posterior sublumbar interbody fusion

The article "Application of Digital Orthopedic Technology in Orthopedic Trauma" was retracted in 2023. Reasons: signs of a paper mill; suspected computer-generated content; unreliable results or conclusions; lack of ethics approval or compliance.

## 5. Conclusion

In this paper, the basic problems of isodigital orthopedic technology in orthopedic assisted therapy were studied, and the main conclusions were as follows:

(1) Within a certain range, the lower the CT scan interval is, the higher the accuracy of 3D reconstruction model is. In the software Mimics, optimal is the fitting option to obtain the best accuracy of the 3D model. Different 3D processing processes produce different reasons for the error of the model. Environmental temperature and other factors have an impact on the model. For the bone, it is not the highest accuracy of the processing method. The shape of the skeleton and the purpose of the printing model should be considered to select the appropriate printing method
(2) In surgical operations, the application of VR 3D printing technology to preoperative simulation can allow doctors to truly observe the structure of the surgical site and provide a reliable basis for clinicians to choose the correct treatment and surgical methods, so as to provide preoperative diagnosis. It can shorten the operation time, minimize the surgical incision, and reduce the incidence of surgical complications, which has very important practical significance
(3) The three-dimensional finite element method was used to model the load applied in the direction of gravity and calculate the force of the normal spine. Effective mechanical support strength can be achieved in posterior sublumbar interbody fusion with pure spinous process lamina. On the basis of the above findings, further study is necessary for the following two questions:
  - When the same 3D printing process is adopted, do different slicing methods (i.e., printing directions) have any influence on the accuracy of the 3D printing model of bone, and what kind of influence will it have
  - The finite element model of the human spine does not consider the ligaments around the vertebral body, and the finite element model can be further improved to analyze the stress changes of the human spine at different postures

## Figures and Tables

**Figure 1:** Application of digital orthopedic technology in orthopedic trauma.

**Figure 2:** Histogram of corresponding point difference of cylinder model under different 3D printing processing technology.

**Figure 3:** Load-deformation curve of the sample.

**Figure 4:** Technical route.

**Figure 5:** Schematic diagram of virtual reality system.

**Table 1:** Comparison of modeling methods.

Grinding method	CT tomography method
Advantages: accurate information of model section geometry and accurate distribution of bone trabecula can be obtained	Advantages: (1) the section geometry is accurate, and it can be quickly and accurately digitized, reducing the error; (2) the integrity of the model is not damaged; (3) the nonuniformity of the section of bone tissue material can be reflected
Disadvantages: (1) the model is destroyed and bone tissue is lost due to cutting; (2) it is difficult to obtain a consistent thickness of the section when the section is very thin; (3) sufficient time is required to prepare the model, and the section geometry is digitized with large error	Disadvantages of nonuniformity of material cross-section: (1) it is difficult to determine the alignment direction of bone trabecula; (2) CT scanning requires multiple channels

The article "Application of Digital Orthopedic Technology in Orthopedic Trauma" was retracted in 2023. Reasons: signs of a paper mill; suspected computer-generated content; unreliable results or conclusions; lack of ethics approval or compliance.

**Table 2:** The gap of polar coordinates under different fitting options when *Z* = 15 mm.

Fit method		Medium	High	Optimal	Custom
Polar gap (d/mm)	Point 1	0.532	0.320	0.051	0.080
	Point 2	0.559	0.388	0.142	0.161
	Point 3	0.572	0.282	0.051	0.002
	Point 4	0.676	0.402	0.122	0.159
	Point 5	0.679	0.490	0.214	0.200
	Point 6	0.563	0.293	0.137	0.143
	Point 7	0.639	0.425	0.198	0.183
	Point 8	0.760	0.420	0.124	0.075
Mean distance		0.631	0.378	0.168	0.164
Standard deviation		0.066	0.077	0.087	0.089

**Table 3:** The gap of polar coordinates under different fitting options when *Z* = 20 mm.

Fit method		Medium	High	Optimal	Custom
Polar gap (d/mm)	Point 1	0.497	0.191	0.068	0.049
	Point 2	0.551	0.209	0.087	0.036
	Point 3	0.535	0.258	0.044	0.045
	Point 4	0.705	0.387	0.131	0.120
	Point 5	0.596	0.286	0.006	0.031
	Point 6	0.511	0.395	0.172	0.174
	Point 7	0.483	0.365	0.149	0.133
	Point 8	0.523	0.374	0.055	0.012
Mean distance		0.545	0.333	0.128	0.121
Standard deviation		0.106	0.084	0.100	0.103

**Table 4:** The gap of polar coordinates under different fitting options when *Z* = 25 mm.

Fit method		Medium	High	Optimal	Custom
Polar gap (d/mm)	Point 1	0.334	0.127	0.059	0.078
	Point 2	0.500	0.232	0.106	0.097
	Point 3	0.62	0.386	0.319	0320
	Point 4	0.599	0.306	0.188	0.175
	Point 5	0.678.	0.359	0.326	0.343
	Point 6	0.631	0.425	0.165	0.174
	Point 7	0.696	0.440	0.159	0.155
	Point 8	0.709	0.442	0.158	0.133
Mean distance		0.630	0.379	0.169	0.165
Standard deviation		0.104	0.102	0.120	0.124

**Table 5:** The gap of polar coordinates under different fitting options when *Z* = 30 mm.

Fit method		Medium	High	Optimal	Custom
Polar gap (d/mm)	Point 1	0.463	0.256	0.099	0.100
	Point 2	0.427	0.119	0.095	0.082
	Point 3	0.582	0.370	0.176	0.176
	Point 4	0.454	0.089	0.083	0.083
	Point 5	0.622	0.407	0.158	0.146
	Point 6	0.558	0.154	0.038	0.045
	Point 7	0.693	0.445	0.256	0.241
	Point 8	0.681	0.375	0.248	0.258
Mean distance		0.625	0.385	0.193	0.194
Standard deviation		0.081	0.120	0.070	0.070

**Table 6:** The gap of polar coordinates under different fitting options when *Z* = 35 mm.

Fit method		Medium	High	Optimal	Custom
Polar gap (d/mm)	Point 1	0.456	0.275	0.128	0.159
	Point 2	0.470	0.200	0.008	0.003
	Point 3	0.660	0.488	0.215	0.234
	Point 4	0.667	0.282	0.001	0.008
	Point 5	0.528	0.500	0.186	0.179
	Point 6	0.662	0.335	0.137	0.114
	Point 7	0.582	0.253	0.073	0.069
	Point 8	0.605	0.311	0.102	0.101
Mean distance		0.597	0.346	0.119	0.123
Standard deviation		0.074	0.124	0.070	0.102

The article "Application of Digital Orthopedic Technology in Orthopedic Trauma" was retracted in 2023. Reasons: signs of a paper mill; suspected computer-generated content; unreliable results or conclusions; lack of ethics approval or compliance.

**Table 7:** The gap of polar coordinates under different fitting options when *Z* = 40 mm.

Fit method		Medium	High	Optimal	Custom
Polar gap (d/mm)	Point 1	0.566	0.416	0.103	0.115
	Point 2	0.614	0.273	0.062	0.165
	Point 3	0.624	0.477	0.201	0.111
	Point 4	0.740	0.465	0.076	0.103
	Point 5	0.658	0.373	0.103	0.105
	Point 6	0.693	0.455	0.175	0.103
	Point 7	0.648	0.416	0.163	0.130
	Point 8	0.655	0.475	0.296	0.298
Mean distance		0.628	0.387	0.148	0.138
Standard deviation		0.048	0.066	0.065	0.056

**Table 8:** Polar distance at different points of the femur of fresh sheep at different heights.

Height		*Z* = 15	*Z* = 20	*Z* = 25	*Z* = 30
Polar gap (d/mm)	Point 1	8.971	8.670	8.503	8.403
	Point 2	8.657	8.922	8.759	8.499
	Point 3	9.502	8.519	8.514	8.966
	Point 4	9.570	8.547	8.981	8.532
	Point 5	8.931	9.285	8.784	8.794
	Point 6	8.895	9.209	8.577	8.637
	Point 7	9.138	8.688	8.351	8.700
	Point 8	8.456	8.453	8.376	8.586
Mean distance		8.892	8.673	8.526	8.553
Standard deviation		0.334	0.276	0.218	0.229

**Table 9:** Finite element model parameters.

Materials	Poisson ratio	Elasticity modulus (MPa)	Density (kg/m^3^)
Cortical bone	0.3	1200	1700
Cancellous bone	0.25	100	1100
Fibre ring	0.45	4.2	1050
Nucleus pulposus	0.5	1.0	

**Table 10:** Titanium alloy, PEEK material parameters.

Name	Directivity	Poisson ratio	Elasticity modulus (MPa)	Density (kg/m^3^)
Medical titanium alloys	Isotropy	0.34	110000	4.5
PEEK	Isotropy	0.1	3800	

**Table 11:** Contact types and properties.

Contact type	Iterations	Normal behavior (separation)	Tangential behavior (sliding)
Bonded	1	Nondisjunction	Nonslip
No separation	1	Nondisjunction	Allow the sliding
No separation	Many times	Clearance allowed	Allow the sliding
Rough	Many times	Clearance allowed	Nonslip
Frictional	Many times	Clearance allowed	Allow the sliding

## Data Availability

The labeled data set used to support the findings of this study is available from the corresponding author upon request.
